The article "Knowledge, Awareness, and Practices (KAP) towards COVID-19 among the marine fishers of Maharashtra State of India: An online cross-sectional Analysis" was published in 2021. Journal: PLoS One.

# Knowledge, Awareness, and Practices (KAP) towards COVID-19 among the marine fishers of Maharashtra State of India: An online cross-sectional Analysis

**DOI:** 10.1371/journal.pone.0261055

**Published:** 2021-12-03

**Authors:** Suhas Wasave, Sangita Wasave, Ketankumar Chaudhari, Prakash Shingare, Bharat Yadav, Sandesh Patil, Bhalchandra Naik

**Affiliations:** 1 Department of Fisheries Resources Economics, Statistics and Extension Education, College of Fisheries, Ratnagiri (Dr. B. S. Konkan Krishi Vidyapeeth, Dapoli, Ratnagiri), Maharashtra, India; 2 Department of Aquaculture, College of Fisheries, Ratnagiri (Dr. B. S. Konkan Krishi Vidyapeeth, Dapoli, Ratnagiri), Maharashtra, India; 3 Associate Dean, College of Fisheries, Ratnagiri (Dr. B. S. Konkan Krishi Vidyapeeth, Dapoli, Ratnagiri), Maharashtra, India; VIT University, INDIA

## Abstract

The knowledge, awareness, and practices (KAP) about COVID-19 among the marine fishers who are engaged in the high-risk occupations and depend on the vulnerable sources of income in the Maharashtra state of India, were investigated to understand the behavioral changes and vulnerability among the respondents because of COVID-19. Data were collected through an online survey from 1^st^ July to 30^th^ July 2020 during the first peak of COVID-19 in the study area by using the questionnaire. Authors based on the latest recommendations by the World Health Organization (WHO) developed the questionnaire and covered the KAP aspects under study. The questionnaire was administered through Google form link and the link was disseminated through social media such as Facebook and What’s App. The completed responses (n = 533) received from the eligible sample, excluding those outsides of the fisher community and duplicate entries were considered for analysis. Appropriate statistical tools were used to analyze the data. Among the respondents, 447 men (83.86%) and 86 women (16.14%), with a mean age of 45.4 years (M = 45.4, SD = 1.18). The results revealed that 70.92% of respondents perceived a low risk of infection because of COVID-19 with M = 1.77 and SD = 0.583, but authors found the perceived severity score high (M = 3.95, SD = 1.21) among the 60.97% of respondents. Around 95% of respondents were aware of the COVID-19, while almost all respondents knew the medium of infection and symptoms of COVID-19. The behavior of respondents towards COVID-19 infection was positive and was following sufficient precautionary measures suggested by WHO to protect themselves from COVID-19 infection. The results of multiple regression analysis revealed that the demographic features of respondents like age, education were significantly contributing to the KAP of the fisher community. The results confirmed the importance of KAP which is reflected in the behavioral responses of the fishers while tackling the COVID-19 pandemic situation. The results regarding the risk perception, severity, KAP about COVID-19 provide a collective understanding of the emerging infectious disease among the marine fishers of Maharashtra state of India.

The article "Knowledge, Awareness, and Practices (KAP) towards COVID-19 among the marine fishers of Maharashtra State of India: An online cross-sectional Analysis" was published in 2021. Journal: PLoS One.

## Introduction

The World Health Organization (WHO) on December 31, 2019, reported the occurrence of an unknown virus [1], which was then renamed by the International Committee as Severe Acute Respiratory Syndrome Coronavirus 2 (SARS-CoV-2) that causes the Coronavirus disease (COVID-19) [2, 3]. Considering unprecedented mortality and morbidity due to COVID-19 and its impact on humankind, WHO declared it as a serious public health emergency of International concern on January 30, 2020 [4]. COVID-19 indicates the symptoms of acute respiratory distress syndrome, septic shock, difficult-to-tackle metabolic acidosis, and bleeding and coagulation dysfunction [5, 6]. The SARS-CoV-2 infected patients are mostly asymptomatic or generally experience mild symptoms that include fever, dry cough, fatigue, myalgia, and dyspepsia [7]. However, some patients in particular the elderly and patients with pre-existing illnesses (like hypertension, cardiac disease, lung disease, cancer, or diabetes) have been identified as potential risk factors for severe disease and mortality [8, 9]. According to some studies [10–12], the infection of COVID-19 mainly occurs through air droplets, close contact with infected persons, especially mucous membranes secretions from nose, mouth, or eyes, contaminated surfaces, digestive tract transmission and also reported that infected person can spread the disease to up to 3 other persons [13].

The countries with high advancement in health systems also faced the worst hit of disease as no proven treatments or reliable vaccines are available to control COVID-19.

Most countries have applied strict prevention and control measures to control the spread of COVID-19, which include general lockdown, obligatory home quarantine, a ban on public gatherings, international flight restrictions, etc. [14]. Also, effective preventive measures have been recommended to the public including hand washing, social distancing, mask-wearing, respiratory hygiene (covering mouth and nose while coughing or sneezing), household ventilation and disinfection, and reduction of interpersonal contacts by avoiding visiting crowded spaces [14, 15].

The little knowledge of disease, negative or casual approach and dangerous practices were the reasons for the spread of COVID-19 infection and subsequent outbreak propagation [16]. The knowledge, attitude, and practices of the community studied in Ethiopia regarding COVID-19 and results revealed that 53.7% of respondents had a negative attitude towards the COVID-19 pandemic [17]. The negative or casual approach of the communities and the relatively disadvantageous categories of society pose a social challenge as they underestimate the COVID-19 risk and keep themselves unaware of symptoms [18]. By implementing the knowledge, awareness, and practice (KAP) studies, it is required to understand the public knowledge, reactions, adherence to, and acceptance of measures that affect psychologically, socially, and physically the daily life of people [19, 20]. The information will improve the awareness level of the citizens and encourage positive attitudes, which could help them in the fight against COVID-19 and similar future threats [19–21].

The article "Knowledge, Awareness, and Practices (KAP) towards COVID-19 among the marine fishers of Maharashtra State of India: An online cross-sectional Analysis" was published in 2021. Journal: PLoS One.

Hitherto, several studies have investigated behavioral responses toward COVID-19 among the general population [22, 23] and in specific populations such as health care workers [24] and college students [25, 26]. In this study, we investigated the KAP towards the COVID-19 outbreak of marine fishers, who are involved in the high-risk occupation and depend on the vulnerable source of income of Maharashtra state in India, which significantly contribute to earn the foreign currency through their capture-based fishing activity. Maharashtra has seven coastal districts spread to 720 Km and 456 fishing villages with a total fisher population of about 4.50 lakhs [27]. For hundred years the fishing communities have been living and working along the coast of Maharashtra and have their way of life and a distinctive culture than the other communities. They live in tight clusters and are known for their unique culture & customs. The traditional fishing sector as, generally of a primitive character, operated by little informed, less organized group of people i.e. fishers and mostly with fewer traditional fishing equipment. Fisher folk remain remained marginalised and far away from the mainstream of development in-spite of the higher socio-economic progress the state has made as a whole. This is a first report aimed to assess the knowledge, awareness, and practices of marine fishers toward COVID-19, and it will probably help the Government and policymakers to initiate effective control measures on the spread of COVID-19 on one of the marginalized categories of society.

## Methodology

### Study design and participants

This is a cross-sectional online survey conducted using a self-administered questionnaire targeting the fisher community of Maharashtra State of India. The male and females from the fisher community of Maharashtra were the target participants for this study. Because of the spread of COVID-19 pandemic and the lockdown situation in the country, a physical and paper-based questionnaire was not practicable. Hence, the questionnaire was designed initially in English and then translated into the local language *Marathi*, and administered through Google form, which was accessible by clicking on a link. Authors through social media such as Facebook and What’s App disseminated the link. The respondents above 18 years old who wish to provide the information were requested to click the link and fill in the information. We were targeting the information on KAP only and anonymity of the respondents was maintained in the final analysis, hence, no separate written or oral consent of respondents, as well as approval of an institutional review board (ethics committee), was taken. Data were collected through an online survey during the first peak of COVID-19 in the study area.

The article "Knowledge, Awareness, and Practices (KAP) towards COVID-19 among the marine fishers of Maharashtra State of India: An online cross-sectional Analysis" was published in 2021. Journal: PLoS One.

### Sample size

The minimum sample size was calculated using the Open Epi-calculator (https://www.openepi.com/SampleSize/SSPropor.htm) [28] to be 471, hypothesizing 97% confidence interval, % frequency of outcome factor in the population 50% +/-5 with a confidence limit of 5% estimated fisher population 0.45 million according to the 2010 census population projection. However, all valid responses received during the period from July 1, 2020, to July 30, 2020 (n = 533) were included in the final analysis excluding those outside of the fisher community, duplicate entries, and incomplete responses.

### Questionnaire design

The questionnaire was developed by authors based on the latest recommendations by the WHO [1, 10, 15, 16]. The questionnaire was pre-tested with 10 respondents from the fisher community for validation and content analysis, and to understand the online Google link access efficiency from the fisher’s point of view. The responses from the pre-test were not included in the final analysis but used to improve the quality of the questionnaire.

The questionnaire was divided into two main sections. The first section was devoted to independent variables under study which included the socio-demographic characteristics of respondents viz. gender, age, education level, health status, health support, and social support especially if they get infected with COVID-19. The second section of the questionnaire was designed to capture information on the dependent variables such as risk perception, awareness about COVID-19, knowledge about the medium of infection and symptoms of COVID-19, precautionary measures, the behavior of fishers if they get infected with COVID-19. The perceived risk of becoming infected with COVID-19 was tested on a three-point scale i.e. High (Score = 3), medium (Score = 2), and low (Score = 1) by asking ’What do you think is the possibility of a COVID-19 infection? And the perceived risk of severity of COVID-19 infection was tested by asking ’What do you think is the severity if COVID-19 infects you?’ with five-point scaling i.e. Very high severity (Score = 5), high severity (Score = 4), moderate severity (Score = 3), low severity (Score = 2), and very low severity (Score = 1). The perceived awareness about COVID-19 was also tested on a three-point scale i.e. High (Score = 3), medium (Score = 2), and low (Score = 1), and the factors related to awareness considered in this study were symptoms, disease spread, precautionary measures and remedies.

The article "Knowledge, Awareness, and Practices (KAP) towards COVID-19 among the marine fishers of Maharashtra State of India: An online cross-sectional Analysis" was published in 2021. Journal: PLoS One.

The perceived knowledge about the medium of infection included six relevant questions to collect information about the topic in question, whereas, to understand the knowledge of symptoms among respondents the various options were given to respondents. The precautionary measures undertaken by respondents to avoid COVID-19 infection were studied by focusing on questions related to (1) preventive measures (e.g., using masks, practicing hand hygiene, avoiding touching mouth and eyes, covering nose and mouth while sneezing and coughing); or (2) social distancing behavior (e.g., reducing the use of public transport, avoid handshakes, keeping distance with persons with fever and cough, avoiding crowded places and postponing or cancelling social events). To check the effectiveness of precautionary measures taken by respondents, the answer was sought by asking ’To what extent do you think each precautionary behavior is an effective way to reduce the risk of COVID-19 infection? And responses were rated on a 5-point Likert-type scale ranging from 1 to 5 with 1 = Not at all effective, 2 = slightly effective, 3 = effective, 4 = highly effective and 5 = extremely effective. The behavior of the respondents was checked if they have symptoms of COVID-19 by asking "what the action they will initiate?" and psychological responses on "how to protect from COVID-19 infection?", belief about prevention of infection, the spread of virus infection, level of protection and time for protection was analyzed. The questions for acquiring information about the medium of infection, knowledge of symptoms, precautionary measures included in the questionnaire, and the options given to respondents to choose only five answers. We gave ten options which included a mixture of correct and wrong answers. Very high knowledge (Score:5) considered among the respondents who had given all correct answers. Four correct answers considered as high knowledge (Score:4), three correct answers as moderate knowledge (Score = 3), two correct answers as low knowledge (Score = 2), and only one correct answer as very low knowledge (Score = 1). If any of the respondents choose all the wrong answers, it will confirm that the particular respondent does not know the subject in question.

The article "Knowledge, Awareness, and Practices (KAP) towards COVID-19 among the marine fishers of Maharashtra State of India: An online cross-sectional Analysis" was published in 2021. Journal: PLoS One.

The reliability of the scale was used to analyze the perceived risk of becoming infected with COVID-19. The perceived awareness about COVID-19 was tested and found to be 0.81. Also, the reliability of scales for analysis of the perceived risk of severity, medium of infection, knowledge of symptoms, precautionary measures was tested and found to be 0.78. For three-point and five-point analysis, the scale was found reliable. We tested the reliability of the scale with Cronbach’s Alpha using the following formula.


$$\propto =\frac{N\bar{c}}{\bar{v}+(N-1)\bar{c}}$$

Here, N = the number of items.

            $\bar{c}$ = average covariance between item-pairs.

    $\bar{v}$ = average variance.

The obtained scores were normalized using following equation

$$\mathrm{Dimension}\;\mathrm{value}=\frac{\mathrm{Actual}\;\mathrm{value}-\mathrm{Minimum}\;\mathrm{value}}{\mathrm{Maximum}\;\mathrm{value}-\mathrm{Minimum}\;\mathrm{value}}$$

Normalized scores were between 0–1, where the perceived risk of becoming infected and perceived awareness considered high (score above 0.66), moderate (score between 0.33–0.66) and low (score between 0–0.33). The perceived risk of severity, medium of infection, knowledge of symptoms, precautionary measures considered very high (score above 0.8), high (score between 0.6–0.8), moderate (score 0.4–0.6), low (score 0.2–0.4), and very low (less than 0.2).

### Data analysis

Fully completed questionnaires extracted from Google Forms and exported to Microsoft Excel for cleaning. Data were summarized using Microsoft Excel and analyzed using the Statistical Package for the Social Sciences (SPSS) software and the OpenEpi. To summarize the obtained data, the demographic characteristics of respondents were subjected to statistics (frequency and percentages). In the present study, the multivariate linear regression analysis was used to examine the association of socio-demographic factors (gender, age, education level) with perceived awareness, perceived knowledge about the medium of infection, perceived knowledge about symptoms, and behavior of fishers if they have symptoms of COVID-19. All statistical analysis was performed in SPSS version 21.0 (IBM Corporation), and a P-value < .05 was considered significant. The precautionary measures taken by respondents to avoid COVID-19 infection were expressed in percentage.

The article "Knowledge, Awareness, and Practices (KAP) towards COVID-19 among the marine fishers of Maharashtra State of India: An online cross-sectional Analysis" was published in 2021. Journal: PLoS One.

## Results

### Socio-demographic characteristics

The demographic characteristics of 533 respondents of the present study revealed that there were 447 men (83.86%) and 86 women (16.14%), with a mean age of 45.4 years (M = 45.4, SD = 1.18) (Table 1). The maximum (31.33%) respondents had secondary-level education, followed by higher secondary (24.20%), while 8.26% of respondent fishers were with graduate-level education, 2.44% had completed their post-graduation and 12.38% studied in Industrial Training Institute to acquaint themselves with skill-oriented learning. 420 (78.8%) and 113 (21.20%) respondents had fishing as a primary and secondary occupation, respectively. The respondents under the study area represented the three major religions viz; Hindu (76.36%), Muslim (15.76%), and Christian (7.88%). The majority of respondents (75.61%) claimed that their health status is good and not had any major health issue since last three years, while 24.39% respondents reported their health status as moderately good as they have undergone health issues like tuberculosis, high sugar, blood pressure, physical injury, etc. Most respondents (60.04%) reported that they would get health support from their families, followed by the government (29.27%) and employer (10.69%) if they get infected with COVID-19 infection. However, the majority of respondents (93.43%) fear that they would not get any social support if they get infected with the COVID-19.

**Table 1:** Socio-demographic factors of respondents (*n* = 533).

Characteristics	Frequency	Percentage
**Gender**	**533**	
Male	447	49.9
Female	86	50.1
**Age groups**	***M* = 45.4**	***SD* = 14.94**
20–30	140	17.7
31–40	143	17.1
41–50	137	19.7
51–60	90	20.5
≥60	23	25.1
**Education**		
Primary	73	13.70
Secondary	167	31.33
Higher Secondary	129	24.20
Industrial Training Institute	66	12.38
Diploma	41	7.69
Graduate	44	8.26
Post Graduate	13	2.44
**Primary occupation**		
Fishing	420	78.80
Service	29	5.44
Business	57	10.69
Agriculture	27	5.07
**Secondary occupation**		
Fishing	113	21.20
Service	107	20.08
Business	164	30.77
Agriculture	149	27.95
**Religion**		
Hindu	407	76.36
Muslim	84	15.76
Christian	42	7.88

### Perceived risk and severity to COVID-19 infection

The respondents were analyzed for the perceived risk of becoming infected with COVID-19 infection was low as only 19.70% of respondents reported that they are under "high" risk of infection (Score = 3), 9.38% claimed to be "medium risk" (Score = 2) and the majority of respondents 70.92% reported "low" risk of COVID-19 infection (Score = 1) with M = 1.77 and SD = 0.583. The perceived severity of COVID-19 infections was found high among fisher respondents (Score = 4) (M = 3.95, SD = 1.21) half of the respondents (50.09%) reported: "very high severity" (Score = 5) of infection. A total of 28.14% had claimed: "moderate severity" (Score = 3), while 6.19% respondents (Score = 2) and 4.69% respondents (Score = 1) reported "low" and "very low severity" of COVID-19, respectively.

The article "Knowledge, Awareness, and Practices (KAP) towards COVID-19 among the marine fishers of Maharashtra State of India: An online cross-sectional Analysis" was published in 2021. Journal: PLoS One.

### Perceived awareness about COVID-19 infection

A total of 58.82% of respondents had high, 36.68% had medium and 4.5% had low awareness about the COVID-19. The channel of information through which the respondents received information about COVID-19 were What’s app (31.71%) followed by Television (20.64%), hospitals (14.63%), family members (6.94%), radio (6.38%), while few respondents were aware by health officer/workers (1.88%). A total of 49.16% of respondents were found aware of the symptoms and 61.16% aware of the precautions to be taken from COVID-19, while 42.78% respondents were aware of the disease spread and about 37.9% respondents were aware of the remedies on COVID-19. The data relating to the awareness of respondents to COVID-19 is summarized in Table 2.

**Table 2:** Perceived awareness about COVID-19 infection.

	Frequency	Percentage
**Level of awareness**		
High	313	58.82
Medium	196	36.68
Low	24	4.50
**Channels of information**		
TV	110	20.64
Radio	34	6.38
What’s app	169	31.71
Family members	37	6.94
friends	46	8.63
Other Social Media	15	2.81
Hospitals	78	14.63
Health officer/ worker	10	1.88
Community leader	34	6.38
**Awareness about COVID-19**		
Symptoms	262	49.16
Disease spread	228	42.78
Precautionary measures	326	61.16
Remedies	202	37.9

The awareness of fishers about COVID-19 was analyzed with multivariate linear regression based on various factors such as symptoms, disease spread, precautionary measures, and remedies (Table 3). The awareness about the symptoms among fishers showed 79% of variance, F (6, 532) = 335.80, adjusted R2 = 0.791, p <0.000. The awareness about disease spread showed the variance of 80%, F (6, 532) = 373.59, adjusted R2 = 0.808, p = 0.000. The awareness about protection measures of COVID-19 is also analyzed. The results revealed the 69% of variance about awareness about protection measures among fishers, F (6, 532) = 201.72, adjusted R2 = 0.694, p = 0.000. The awareness about the remedies on COVID-19 showed 78% variance, F(6, 532) = 326.56, adjusted R2 = 0.786, p = 0.000. As shown in Table 3, the age was negative and significant in predicting awareness about symptoms, disease spread, precautionary measures, and remedies. Similarly, the education was also negative and significant in awareness about symptoms, disease spread, and precautionary measures, but it was negative and non-significant in predicting awareness about remedies.

The article "Knowledge, Awareness, and Practices (KAP) towards COVID-19 among the marine fishers of Maharashtra State of India: An online cross-sectional Analysis" was published in 2021. Journal: PLoS One.

**Table 3:** Results of multivariate linear regression analysis of perceived awareness about COVID-19 infection.

**Variables**	Symptoms					Disease spread				
	**B (95% CI)**	**Std. Error**	**Beta**	**t**	***p-*Value**	**B (95% CI)**	**Std. Error**	**Beta**	**t**	***p-*Value**
(Constant)	1.452 (1.44–1.47)	.065		22.218	.000	1.347 (1.24–1.45)	.062		21.746	.000
Gender	-.195 (-0.53–0.14)	.086	-.144	-2.266	.024	-.018 (-.32–0.36)	.082	-.013	-.217	.828
Age group	-.361 (-0.22–0.51)	.029	-.849	-12.521	.000	-.110 (-0.02–0.24)	.027	-.262	-4.033	.000
Education	-.179 (-0.30–0.67)	.025	-.559	-7.143	.000	-.128 (-0.03–0.23)	.024	-.404	-5.387	.000
**Variables**	Precautionary measures					Remedies				
	**B (95% CI)**	**Std. Error**	**Beta**	**t**	***p-*Value**	**B (95% CI)**	**Std. Error**	**Beta**	**t**	***p-*Value**
(Constant)	1.556 (1.40–1.71)	.077		20.171	.000	1.342 (1.17–1.52)	.064		20.948	.000
Gender	-.123 (-0.47–0.22)	.102	-.093	-1.214	.225	-.086 (-0.43–0.26)	.084	-.066	-1.020	.308
Age group	-.231 (-0.042–0.04	.034	-.557	-6.795	.000	-.141 (-0.03–0.25)	.028	-.342	-4.988	.000
Education	-.159 (-0.32–0.00)	.030	-.509	-5.375	.000	-.015 (-0.10–0.07)	.025	-.047	-.596	.552

### Perceived knowledge about vulnerable age group and medium of infection of COVID-19

The highest (60.60%) of respondents revealed that both children (<10) and old persons (>60) are vulnerable to the COVID-19 infection, whereas 29.27 and 10.13% of respondents believed that only the aged persons and children are vulnerable to the COVID-19 infection, respectively. When enquired about the medium of infection of COVID-19 with respondents, we received multiple responses. The maximum no. of respondents (55.22%) reported that contact with an infected person is the primary medium of infection, while 45.48% claimed that spit/slim of infected person is medium of COVID-19 infection. The other mediums of infection mentioned are sex with an infected person (33.48%), unknowingly touching infected surfaces (31.60%), contact with infected animals (23.72%), and consumption of stale food (10.50%) (Table 4).

**Table 4:** Perceived knowledge about vulnerable age group and medium of infection of COVID-19.

	Frequency	Percentage
**Most vulnerable to COVID-19**		
Children below 10 years age	54	10.13
Old persons above 60 years age	156	29.27
Both children and old persons	323	60.60
**Medium of infection of COVID-19**		
In contact with infected person	294	55.22
Spit/slim of infected person	242	45.48
Sex with infected person	178	33.48
Unknowingly touching the infected surface	168	31.60
In contact with infected animals	136	23.72
Consumption of stale food	56	10.50

The knowledge of fishers about COVID-19 was analyzed with multivariate linear regression and is depicted in Table 5. The contact with an infected person is considered as a medium of infection, and it has a variance of 76%, F(6,526) = 296.23, adjusted R2 = 0.769, p = 0.000. The spit/slim of the human being is also considered as medium of infection with variance of 80%, F (6, 526) = 362.51, adjusted R2 = 0.803, p = 0.000. The sex with the infected person was also one of the mediums of infection and has a variance of 75%, F(6, 526) = 279.46, adjusted R2 = 0.758, p = 0.000. The unknowingly touching the infected surface was also one of the mediums of infection of COVID-19 known to respondents, which has 75% variance, F(6, 526) = 274.36, adjusted R2 = 0.755, p = 0.000. Similarly, contact with infected animals is also the medium of infection which has a variance of 76%, F(6, 526) = 288.31, adjusted R2 = 0.764, p = 0.000. The consumption of stale food is one medium of infection as described by the respondents with 37% variance, F(6, 526) = 51.63, adjusted R2 = 0.363, p = 0.000. In predicting the perceived knowledge about the medium of infections, gender and age showed a negative but significant impact. The education (β = 0.058, p < 0.022) had shown a significant positive impact on unknowingly touching the infected surface as the medium of infection. However, education showed either a negative significant or non-significant impact on the knowledge of other variables.

The article "Knowledge, Awareness, and Practices (KAP) towards COVID-19 among the marine fishers of Maharashtra State of India: An online cross-sectional Analysis" was published in 2021. Journal: PLoS One.

**Table 5:** Results of multivariate linear regression analysis of perceived knowledge about medium of infection of COVID-19.

**Variables**	**Contact with infected person**					**Spit/slim of the human**					**Sex with infected person**				
	**B (95% CI)**	**Std. Error**	**Beta**	**t**	***p-*Value**	**B (95% CI)**	**Std. Error**	**Beta**	**t**	***p-*Value**	**B (95% CI)**	**Std. Error**	**Beta**	**t**	***p-*Value**
(Constant)	1.584 (1.51–1.66)	.068		23.198	.000	1.323 (1.26–1.39)	.063		20.947	.000	1.298 (1.06–1.53)	.066		19.592	.000
Gender	-.290 (-0.01–0.57)	.090	-.216	-3.227	.001	-.044 (-0.16–0.72)	.083	-.032	-.525	.600	-.175 (-0.48–0.13)	.087	-.137	-2.010	.045
Age group	-.449 (-0.28–0.62)	.030	-1.060	-14.886	.000	-.197 (0.03–0.37)	.028	-.465	-7.071	.000	-.232 (-0.04–0.42)	.029	-.578	-7.946	.000
Education	-.133 (-0.29–0.03)	.026	-.418	-5.087	.000	-.230 (-0.07–0.39)	.024	-.723	-9.527	.000	.036 (-0.14–0.21)	.025	.118	1.408	.160
**Variables**	**Unknowingly touching the infected surface**					**Contact with infected animal**					**Consumption of stale food**				
	**B (95% CI)**	**Std. Error**	**Beta**	**t**	***p-*Value**	**B (95% CI)**	**Std. Error**	**Beta**	**t**	***p-*Value**	**B (95% CI)**	**Std. Error**	**Beta**	**t**	***p-*Value**
(Constant)	1.278 (1.02–1.54)	.066		19.454	.000	1.193 (0.85–1.54)	.061		19.716	.000	.269 (-0.29–0.83)	.070		3.843	.000
Gender	-.214 (-0.53–0.10)	.086	-.170	-2.474	.014	-.297 (-0.02–0.58)	.080	-.252	-3.735	.000	.123 (-0.30–0.55)	.092	.148	1.335	.182
Age group	-.272 (-0.07–0.47)	.029	-.687	-9.377	.000	-.351 (-0.18–0.52)	.027	-.946	-13.152	.000	.039 (-0.24–0.32)	.031	.148	1.256	.210
Education	.058 (-0.12–0.24)	.025	.194	2.289	.022	.117 (-0.04–0.28)	.023	.419	5.046	.000	-.197 (-0.44–0.05)	.027	-1.003	-7.356	.000

The article "Knowledge, Awareness, and Practices (KAP) towards COVID-19 among the marine fishers of Maharashtra State of India: An online cross-sectional Analysis" was published in 2021. Journal: PLoS One.

### Perceived knowledge about symptoms of COVID19

The respondents narrated about multiple symptoms of COVID-19. Around half of the respondents (47.28%) reported cough is one symptom of COVID-19 with variance of 79%, F(6,526) = 336.53, adjusted R2 = 0.791, p = 0.000. A total of 42.78% claimed that fever is the symptom of COVID-19. The knowledge of symptoms of COVID-19 regarding fever showed the variance of 80%, F(6,526) = 370.90, adjusted R2 = 0.807, p = 0.000. A total of 33.40% respondents reported difficulty in breathing as a symptom which has a variance of 75%, F(6, 526) = 279.46, adjusted R2 = 0.758, p = 0.000. 15.76% stated that sore throat is also a symptom of COVID-19 which has a variance of 50%, F(6, 526) = 93.024, adjusted R2 = 0.509, p = 0.000. Very few respondents informed that diarrhea (0.38%), vomiting (0.94%) and body pain (3%) were also symptoms of COVID-19 (Tables 6 and 7). The gender has negative and non-significant in predicting the cough, fever, sore throat as symptoms of COVID-19 and it was negatively significant in predicting difficulty in breathing as symptoms of COVID-19. Table 7 also reveals age as negative significant in predicting the cough, fever, and difficulty in breathing as symptoms of COVID-19. The education also had a significant and negative impact in predicting the variables such as cough, fever, and sore throat as symptoms of COVID-19.

**Table 6:** Perceived knowledge about symptoms of COVID-19.

Symptoms	Frequency	Percentage
Fever	228	42.78
Cough	252	47.28
Difficulty in breathing	178	33.40
Headache	8	1.50
Sore throat	84	15.76
Diarrhoea	2	0.38
vomiting	5	0.94
Body pain	16	3.00

**Table 7:** Results of multivariate linear regression analysis of perceived knowledge of symptoms of COVID-19.

**Variables**	Cough					Fever				
	**B (95% CI)**	**Std. Error**	**Beta**	**t**	***p-*Value**	**B (95% CI)**	**Std. Error**	**Beta**	**t**	***p-*Value**
(Constant)	1.344 (1.084–1.604)	.062		21.610	.000	1.391 (1.131–1.651)	.065		21.324	.000
Gender	-.018 (-0.46–0.10)	.082	-.013	-.218	.827	-.123 (-0.40–0.16)	.086	-.091	-1.436	.152
Age group	-.115 (-0.28–0.05)	.027	-.274	-4.203	.000	-.284 (-0.11–0.46)	.029	-.667	-9.846	.000
Education	-.137 (-0.29–0.02)	.024	-.433	-5.756	.000	-.203 (-0.04–0.36)	.025	-.636	-8.136	.000
**Variables**	Difficulty in breathing					Sore throat				
	**B (95% CI)**	**Std. Error**	**Beta**	**t**	***p-*Value**	**B (95% CI)**	**Std. Error**	**Beta**	**t**	***p-*Value**
(Constant)	1.298 (1.038–1.558)	.066		19.592	.000	.530 (0.27–0.79)	.073		7.266	.000
Gender	-.175 (9–0.48–0.13)	.087	-.137	-2.010	.045	.091 (-0.30–0.48)	.096	.092	.946	.345
Age group	-.232 (-0.04–0.42)	.029	-.578	-7.946	.000	.015 (-0.24–0.27)	.032	.049	.475	.635
Education	.036 (0.18–0.54)	.025	.118	1.408	.160	-.152 (-0.38–0.07	.028	-.652	-5.447	.000

The article "Knowledge, Awareness, and Practices (KAP) towards COVID-19 among the marine fishers of Maharashtra State of India: An online cross-sectional Analysis" was published in 2021. Journal: PLoS One.

### Behavior of respondents if they have symptoms of COVID19

The respondents were asked if they have symptoms of COVID-19, what action they will initiate? Table 8 depicted the actions of the respondents. About half of the respondents (48.78%) reported that they will go to the hospital/health unit for further check-ups. 32.27% of respondents declared that they will quarantine themselves for early recovery and avoid the further probable spread of disease. About 12.01% and 6.75% of respondents found a casual approach and said that they will visit a neighborhood nurse and look for advice from an experienced relative, respectively.

**Table 8:** Behavior of respondents if they have symptoms of COVID-19.

Actions	Frequency	Percentage
Look for a more experienced relative for advise	36	6.75
Go to hospital /health unit	260	48.78
Visit to the neighborhood nurse	64	12.01
Quarantine himself	172	32.27

### Precautionary measures taken to avoid COVID19 infection

The Standard Operational Protocol (SOP) of WHO as a precautionary measure to avoid COVID-19 infection was found followed by the majority of fishers of Maharashtra. Table 9 revealed that about 47.65% of respondents used masks, 46.53% respondents avoided crowding places, 45.03% of respondents washed hands for at least 20 seconds each time, 44.28% of respondents avoid touching mouth and eyes, 42.40% of respondents used sanitizer for washing hands, 39.77% of respondents know to cover nose and mouth while sneezing and coughing, 39.40% avoid handshakes with others, 37.52% respondents keep themselves away from persons with fever and cough, 30.39% respondents taking effort to improve their immune system, 18.39% avoiding contact with animals and any surface and 11.26% respondents take care of themselves by drinking clean and warm water.

**Table 9:** Knowledge of respondents about precautionary measures to be taken to avoid COVID-19 infection.

Precautionary measures	Frequency	Percentage
Washing hands for 20 seconds each time	240	45.03
Use of mask	254	47.65
Use of sanitizer for washing hands	226	42.40
Avoid hand shake	210	39.40
Maintain social distancing	218	40.90
Avoid crowding places	248	46.53
Improve immune system	162	30.39
Cover nose and mouth while sneezing and coughing	212	39.77
Do not touch mouth and eyes	236	44.28
Keep away from persons with fever and cough	200	37.52
Avoid contact with animals and surface	98	18.39
Drink clean and warm water	60	11.26

The article "Knowledge, Awareness, and Practices (KAP) towards COVID-19 among the marine fishers of Maharashtra State of India: An online cross-sectional Analysis" was published in 2021. Journal: PLoS One.

## Discussion

The results provide comprehension about the knowledge, attitude, and practices related to the COVID-19 pandemic among the marine fishers of Maharashtra State of India. Most participants reported the perceived severity of COVID-19 virus infections as high; however, the respondents claimed the risk of becoming infected with COVID-19 virus infection was low as the respondents found taking precautions themselves, regardless of the recommendations by the Government and health agencies to reduce the risk of COVID-19 infections. The psychological response of the respondents under study regarding the perceived severity and risk found inversely proportional and we can attribute this to the knowledge, attitude, and practices level of respondents. However, perceived severity is considered as playing an important role when individuals have already been diagnosed with certain diseases [29].

The perceived awareness about COVID-19 was high (58.82%) among the respondents, and they were aware of basic information related to symptoms, disease spread, and preventive measures through social media, television, hospitals, family members, radio, etc. The rate of awareness among fishers about symptoms, disease spread, and preventive measures of COVID-19 was substantial than expected, thus we have denoted it as high. WHO declared COVID-19 as an urgent public health emergency of international concern on January 30, 2020, and we conducted the present survey in July 2020, immediately after the spread of COVID-19, which was the peak in India. In this survey, we found almost half of the respondents were aware of the symptoms, disease spread, and preventive measures of COVID-19. Since the fishers spend most of their time at sea, away from the mainstream of information sources, we deliberated the awareness in this study high. Similar results reported mentioning that the most used information sources about COVID-19 were television programs, websites as local/national networks, newspapers, and social networks [30–32]. In the initial phase of the evolution of the COVID-19 pandemic, social media and newspapers were full of information about COVID-19. The Central Government via Prasar Bharati TV and radio channel provided valuable information to the people. However, most of the other sources of information comprising social media were unreliable and busy in supplying false and scary information about the COVID-19 pandemic, which gave rise to panic and havoc situations all over the country. Though social media was the primary source of information to most people, it was also a primary source of misinformation and falsehood [33]. Similarly, many researchers showed agreement with this and pointed out the danger of fake news and misinformation on social media [34–36]. On the other hand, the majority of citizens worldwide acquire information received through social media without checking its source [29, 37–39]. Despite that, we found most of the respondents in this study with knowledge about the COVID-19. Similar results were reported [32] mentioning that the majority of the respondents (61.6%) had good knowledge of the disease. The survey undertaken in Bangladesh revealed that 48.3% of participants had more accurate knowledge, 62.3% had more positive attitudes, and 55.1% had more frequent practices regarding COVID-19 prevention [40].

The article "Knowledge, Awareness, and Practices (KAP) towards COVID-19 among the marine fishers of Maharashtra State of India: An online cross-sectional Analysis" was published in 2021. Journal: PLoS One.

In present study, we found moderate knowledge (37.9%) about the genuine medium of infections of COVID-19 among the respondents. The investigation undertaken in Addis Ababa, Ethiopia [41] reported similar results mentioning that 58.6% of the respondents had moderate knowledge and 37.2% respondents had excellent knowledge about COVID-19. The respondents acquired this information from the health agencies, private hospitals, and extensive awareness campaigns on social media, television, radio, newspapers by Government. The majority of the respondents had good knowledge about the transmission mode and symptoms of COVID-19 and they got information mainly through mass media [42, 43].

The direct contacts with an infected person, spit/slim of infected person, sex with an infected person, unknowingly touching infected surfaces were the correct medium of infections informed by respondents. We can attribute this to the reliable sources of information received from respondents. However, the consumption of stale food is a medium of infection of COVID-19, which was informed by few respondents. This is because of excessive reliance on social media, which was contributed significantly to misinformation. Also, the socio-demographic factors such as education, age were significant while in understanding the medium of infection among respondents. The educated, as well as elderly respondents, were with knowledge about the medium of disease. In the present study, the respondents reported symptoms of COVID-19 are fever, cough, difficulty in breathing, headache, sore throat, diarrhea, vomiting, and body pain. They received this knowledge of symptoms from social media, television, radio, hospitals, health workers, relatives, family members, friends, etc. The few sources of information which contributed to the knowledge about symptoms of COVID-19 may not be reliable i.e. social media, relatives, family members, friends; hence, the vomiting and body pain were also known as symptoms of COVID-19, which are not proven scientifically [44]. The study on COVID-19 assessment of knowledge and awareness in Indian society revealed that considerable numbers of respondents were aware of the common symptoms of COVID-19 [45].

The article "Knowledge, Awareness, and Practices (KAP) towards COVID-19 among the marine fishers of Maharashtra State of India: An online cross-sectional Analysis" was published in 2021. Journal: PLoS One.

The findings of the present study had an agreement with a study undertaken by other researchers reporting that the most common symptoms include fever, cough, dyspepsia, myalgia, and fatigue [46–51]. Other symptoms are anorexia, nausea, and diarrhoea [46, 47, 49, 50, 52, 53]. Further, the respondents were found aware of the seriousness of these symptoms to old-age persons (above 65) and children (age below 10). Besides, the respondents informed that persons with cardiovascular problems, chronic lung disease, hypertension, diabetes, and obesity are bearing a high risk of being infected with the COVID-19 virus. These findings agreed with the results reported by [49, 52, 54, 55].

The behavior of respondents was found positive in the situation if they have symptoms of COVID-19. The majority of respondents reported they would go to the hospital/health unit and quarantine themselves for early recovery and to avoid further spread of COVID-19 as a carrier from them. This agrees with the findings of the present study mentioning that most of the respondents had perceived awareness, the perceived knowledge about the medium of infection, and symptoms of COVID-19. Only a few respondents (18.76%) were with a casual approach and reported that they would visit the neighborhood nurse or look for advice from experienced relatives. This behavior is also of serious concern and affects the overall image of the respondents under study i.e. marine fishers.

We found most of the respondents serious about the future possibility of COVID-19 infections, and therefore, they will take a few precautionary measures to protect themselves. We can attribute this to adequate knowledge about COVID-19 and its preventive measures declared by WHO [43]. The majority (96.7%) of the participants agreed ’COVID-19 is a dangerous disease’, almost all (98.7%) participants wore a face mask in crowded places, 98.8% agreed to report a suspected case to health authorities, and 93.8% implemented washing hands with soap and water [41]. Hand washing and wearing of face masks have long been regarded as significant preventive habits in the daily life of the public since they proved them to be efficacious in preventing influenza and SARS [41, 56, 57]. According to the findings of [58], 64.6%-86.6% of respondents were practicing five major preventive behaviors. Further, the study reported that over 80% of respondents had been in favor of increased hand washing and face mask-wearing and decreased time spent in crowds, showing that basic protective behaviors against COVID-19 had taken root among respondents. The study [59] revealed that 98, 95 and 77% of the population knew the main preventive measures of the disease spread (hand washing, social distancing, and masks) and further recommended transferring this knowledge into practice to control the disease. In connection to this recommendation [60], added that the health education intervention would be more effective if it targets certain demographic groups, older adults and rural people at the grass-root level who are more likely to have poor knowledge, negative attitudes, and inappropriate preventive practices towards COVID-19.

The article "Knowledge, Awareness, and Practices (KAP) towards COVID-19 among the marine fishers of Maharashtra State of India: An online cross-sectional Analysis" was published in 2021. Journal: PLoS One.

We found the respondents under the present study were psychologically strong and concerning COVID-19 infections. Half of the respondents knew to protect them from disease infection and almost half of the respondents believed that disease infection can be prevented as they know how does coronavirus infection spreads, what are the symptoms of it, and the time required for disease infection. The psychological responses are essential for behavioral responses and can significantly influence the level of public preparedness in a public health emergency such as the COVID-19 pandemic [59].

## Conclusions

The COVID-19 pandemic has affected the social, cultural, economic life of human beings and emerged as one challenge to the medical, psycho-social, political, economic life of countries around the globe. The disbelief that arises because of misinformation about the COVID-19 significantly affected the psychological mind-set of individuals and communities. This study is one of the first conducted among the people of society who are engaged in the high-risk occupations and depend on the vulnerable sources of income i.e. marine fishers of Maharashtra state of India, to understand the KAP regarding the COVID-19. The study confirms that the respondents despite their underprivileged status compared to other societies, had in-depth knowledge of COVID-19 symptoms, its precautionary measures to be taken and remedies. The respondents also had positive behavior if they become infected with COVID-19. The respondents found accessing the knowledge related to COVID-19 from various channels of information. The results regarding the risk perception, awareness, knowledge, attitude, practices about COVID-19 provide a collective understanding of the emerging infectious disease among the marine fishers. The socio-demographic factors such as age, education were found to contribute significantly to the knowledge, attitude, and practices of the respondents regard to COVID-19.

The article "Knowledge, Awareness, and Practices (KAP) towards COVID-19 among the marine fishers of Maharashtra State of India: An online cross-sectional Analysis" was published in 2021. Journal: PLoS One.

## Limitations

This study has a few limitations. First, the study was conducted through online mode. We have included respondents who have access to social media networks in this study, hence it would not be reflected the opinions of the whole fisher population of Maharashtra, India. Second, the respondents might have given socially desirable responses. Third, we perform the present study with tools to assess the knowledge, awareness, and practices of the respondents based on the previous studies by the other researchers [60] adhering to the locale of the study and pandemic situation.
